This article has been retracted.

# Extracellular Vesicles Derived from Lung Cancer Cells Induce Transformation of Normal Fibroblasts into Lung Cancer-Associated Fibroblasts and Promote Metastasis of Lung Cancer by Delivering lncRNA HOTAIR

**DOI:** 10.1155/2022/3805013

**Published:** 2022-10-11

**Authors:** Xiaoxuan Zhang, Yan Zhang, Xin Qiu, Jing Cai, Zhenzhou Yang, Fangzhou Song

**Affiliations:** ^1^Molecular Medicine and Cancer Research Center, Chongqing Medical University, Chongqing 400016, China; ^2^Department of Biochemistry and Molecular Biology, Chongqing Medical University, Chongqing 400016, China; ^3^Department of Cancer Center, The Second Affiliated Hospital, Chongqing Medical University, Chongqing 400010, China

## Abstract

Human lung cancer (LC) cells A549/H358, normal lung epithelial cells BEAS-2B, and lung normal fibroblasts (NFs) were cultured, followed by transfection of H358 cells with HOTAIR shRNA. Extracellular vesicles (EVs) extracted from H358 cells were identified. The internalization of Dil-labeled-EVs by NFs was tested, and protein levels of cancer-associated fibroblast (CAF) surface markers, inflammatory cytokines, cell proliferation, invasion, and migration, and lncRNA HOTAIR levels were determined. A549 cells were cultured in an H358-EVs-treated conditioned medium of NFs (NFCM), followed by intravenous injection of A549 cells into nude mice. The lesions and Ki-67-positive cells in lung tissues were measured. The results showed that tumor cell-derived EVs (T-EVs) motivated the transformation of NFs into CAFs. Specifically, EVs can be internalized by NFs, and the protein levels of CAF surface markers and inflammation levels were elevated in H358-EVs-treated NFs. The proliferation, invasion, and migration of A549 cells cultured in T-EVs-treated NFCM were increased. H358-EVs carried HOTAIR into NFs and promoted the transformation of NFs into CAFs. Inhibition of HOTAIR partially reversed the promoting effect of H358-EVs on the transformation of NFs into CAFs and invasion and migration of LC cells. T-EVs promoted metastasis of LC *in vivo* by transforming NFs into CAFs.

## 1. Introduction

Lung cancer (LC) remains one of the most deadly malignancies, accounting for one-fifth of all cancer deaths [1]. Meanwhile, LC is a highly heterogeneous disease that occurs in a variety of anatomical sites throughout the respiratory tract [2]. It has been reported that repeated damage in lung cells caused by various environmental factors leads to lung tissue damage, thereby inducing genetic and epigenetic changes as well as global transcriptome changes [3]. Moreover, long-term changes at the DNA level lead to abnormal activation of multiple oncogenic pathways and inactivation of tumor suppressor pathways, as well as irreversible changes in cell function, which ultimately induce precancerous lesions, including dysplasia and clonal plaques (early stage of LC) [4, 5]. In addition, the growth of tumor cells is provoked by additional alterations, such as co-occurrence of mutations, metabolic changes, and immune evasion, which eventually leads to the invasion and metastasis of tumor cells (advanced LC) [6, 7]. Since the clinical symptoms of early LC are not obvious and difficult to identify, most patients with LC are commonly diagnosed at an advanced stage [8, 9]. In recent years, despite progress in the treatment options, the prognosis of patients with advanced LC is still poor [10]. Moreover, due to delayed diagnosis, the 5-year survival rate of LC is less than 5%, which is much lower than other cancer patients [11, 12]. More importantly, LC has high incidence and high metastasis rates and has become the number one killer in all cancer [13, 14]. Currently, the tumor microenvironment (TME) associated with LC progression has been a hot topic in the study of effective prognosis and therapeutic targets of LC [15].

TME consists of cancer cells, immune cells, stromal cells, and cytokines, among which stromal cells are composed of cancer-associated fibroblasts (CAFs), immune cells, and vascular endothelial cells [16–19]. What is noteworthy is that normal fibroblasts (NFs) are essential in tissue homeostasis under normal conditions and mediate proper cellular communication and functions; additionally, NFs can be activated by cancer-secreted factors, and these activated NFs are considered CAFs [20]. CAFs are the most important stromal component of the TME, encouraging tumor growth and metastasis [21]. Specifically, CAFs secrete growth factors, chemokines, matrix metalloproteases, and extracellular matrix (ECM) to regulate tumor growth, angiogenesis, and recruitment of bone marrow-derived cells, thereby promoting metastasis [22–24]. Additionally, CAFs, characterized by expression of alpha-smooth muscle actin (*α*-SMA) and fibroblast activation protein- (FAP-) *α*, are the most representative stromal cells in the TME, providing nutrients for tumor development and metastasis by interacting with tumor cells [25, 26]. Meanwhile, CAFs can regulate the inflammatory microenvironment by expressing proinflammatory genes such as interleukin (IL)-1*β*, IL-6, IL-8, TGF-*β*, CXCL12, and collagen [27–29]. Importantly, CAFs produce a large amount of IL-6 in the TME, induce epithelial-mesenchymal transition through the IL-6/STAT3 pathway, and enhance the metastasis potential of LC [30]. Hence, elucidating the regulatory mechanism of CAF activity may lay a theoretical foundation for new therapies targeting TME.

External vesicles (EVs) are a group of heterogeneous cell-derived vesicles composing of small exosomes and large microvesicles [31]. It has been verified that tumor cell-derived EVs (T-EVs) regulate the motivation of CAF phenotypes in the TME, which can be mediated by several EV cargoes such as miRNAs, proteins, mRNAs, and long noncoding RNA (lncRNAs) [32]. LncRNAs, a subgroup of ncRNAs with a length of more than 200 nt and without protein-coding function, have been recognized for their mediating effects on the development of a variety of tumors [33–35]. Transforming growth factor-*β* (TGF-*β*), fibroblast growth factor 2, epidermal growth factor, hypoxia, reactive oxygen species, and ncRNAs are the key regulators of fibroblast activation [36, 37]. With the development of sequencing technologies such as gene chips and next generation sequencing, lncRNAs are identified to play a role as a transmitter between tumor cells and CAFs and participate in the activation of NFs to CAFs [21]. In addition, tumor cells and CAFs can communicate more directly through Exos-carrying lncRNAs, and Exos released by cancer cells can also promote the transformation and activation of CAFs [32]. Meanwhile, Exos secreted by tumors may be optimal lncRNA carriers to provide a mechanism for lncRNA transport to the TME [38]. It has been reported that the tumor-derived exosomal lncRNA POU3F3 promotes the resistance of esophageal squamous cell carcinoma cells to cisplatin by inducing the transformation of fibroblasts into CAFs [39].

LncRNA HOTAIR has been reported to be highly expressed in LC and promotes cisplatin resistance in non small-cell LC cells [21, 40], thus being as a marker of abnormal regulation of the LC cell cycle [41]. Moreover, HOTAIR knockdown could partially reverse the promoting effect of Caveolin-1 on cell viability and invasiveness, and HOTAIR may be a new therapeutic target for LC [42]. Besides, inhibition of HOTAIR inhibits LC cell growth [43]. In light of the above literature, we speculate that T-EVs may facilitate the activation of CAFs by carrying HOTAIR, thus promoting the metastasis of LC. Nevertheless, it remains unclear whether LC cells activate CAFs by secreting EV-carrying HOTAIR. This study set out to explore the underlying mechanism of LC cell-derived EVs affecting the invasion and metastasis of LC by accelerating the activation of CAFs.

## 2. Materials and Methods

### 2.1. Ethics Statement

All animal experiments were conducted under the guidelines and ratified by the Animal Care and Use Committee of Chongqing Medical University. The animal experiments were conducted on the principle of minimized animal number and the least pain.

### 2.2. Cell Culture

Human LC cell lines A549 and H358, normal lung epithelial cell line BEAS-2B (ATCC, Rockville, MD, USA), and lung NFs (Procell, Wuhan, China) were subcultured in DMEM (Gibco, NY, USA) supplemented with 10% fetal bovine serum (FBS), 100 U/mL penicillin, and 100 *μ*g/mL streptomycin in a humidified incubator at 37°C with 5% CO_2_. The medium was replaced every 2-3 days.

### 2.3. Isolation, Identification, and Grouping of EVs

When H358/BEAS-2B cells reached about 80% confluence, they were cultured in an EV-free medium for 48 hours, followed by centrifugation at 2000 g for 10 minutes at 4°C to collect the supernatant, and centrifugation at 10000 g for 40 minutes at 4°C, and then the supernatants were collected. Afterwards, the samples were centrifuged at 110000 g at 4°C for 90 minutes followed by supernatant removal. Then, the precipitates were washed with phosphate-buffered solution (PBS) and centrifuged at 110000 g at 4°C for 90 minutes, and the supernatants were discarded to obtain EVs. Lastly, the EVs resuspended with PBS were preserved at −80°C.

EVs were identified by the following methods: (A) the morphology of EVs was observed by a transmission electron microscope (TEM); (B) the particle size distribution of EVs was analyzed by nanoparticle tracking analysis (NTA); (C) Western blotting was employed to measure the level of positive markers, CD9 and CD81, and negative marker Calnexin on EV surface; (D) cell supernatant treated with EV inhibitor GW4869 (10 nm, Sigma-Aldrich, MO, USA) for 2 hours was served as the control (GW) [44]. The total protein content of EVs was determined with the bicinchoninic acid (BCA) kits (23225, Thermo Fisher, Shanghai, China) according to the instructions, and protein content was considered the standard when EVs were used.

EVs were grouped as follows: the GW (H358-GW/BEAS-2B-GW) group, the EVs (H358-EVs/BEAS-2B-EVs) group, the H358-EVs+Rnase group (EVs treated with Rnase), the H358-EVs+Rnase+sodium-dodecyl-sulfate (SDS) group (treated with Rnase and SDS), the H358-EVs-si-negative control (NC) group (EVs were extracted after transfection of H358 cells with HOTAIR scramble), and the H358-EVs-si-HOTAIR group (EVs were extracted after transfection of H358 cells with HOTAIR shRNA). HOTAIR shRNA and HOTAIR scramble (GenePharma, Shanghai, China) were transfected into cells using Lipofectamine 2000 (Invitrogen, CA, USA).

### 2.4. NF Treatment and Grouping

NFs were cultured to the third generation. When the cell confluence reached about 90%, the cells were treated and grouped as follows: (1) the NFs group: without any treatment; (2) the EVs^BEAS-2B^ group: treated with BEAS-2B-EVS (50 *μ*g) for 6 hours [45]; (3) the GW^BEAS-2B^ group: treated with an equal amount of BEAS-2B-GW for 6 hours; (4) the EVs^H358^ group: treated with H358-EVs (50 *μ*g) for 6 hours; (5) the GW^H358^ group: treated with the same amount of H358-GW for 6 hours; (6) the EVs^H358-si-HOTAIR^ group: treated with H358-EVS-si-HOTAIR (50 *μ*g) for 6 hours; and (7) the EVs^H358-si-NC^ group: treated with H358-EVs-si-NC (50 *μ*g) for 6 hours.

### 2.5. Treatment and Grouping of A549 Cells

When NFs reached about 50% confluence, the medium was supplemented and incubated for 48 hours. After centrifugation at 200 g for 10 minutes, the collected supernatants were NFs-conditioned culture medium. A549 cells were cultured in a mixture of a conditioned medium of NFs (NFCM) and A549 cell medium in a volume ratio of 1 : 2 for 24 hours [45].

A549 cells were allocated into the following 4 groups: the A549+GW^H358^ group (cultured in NFCM treated with H358-GW), the A549+EVs^H358^ group (cultured in NFCM treated with H358-EVs), the A549+EVs^H358-si-NC^ group (cultured in NFCM treated with H358-EVs-si-NC), and the A549+EVs^H358-si-HOTAIR^ group (cultured in NFCM treated with H358-EVs-si-HOTAIR).

### 2.6. Immunofluorescence Assay

EVs were labeled with Dil dye (Invitrogen) and coincubated with NFs for 24 hours. NFs were rinsed twice with PBS, fixed with 4% paraformaldehyde, counterstained with 4′,6-diamidino-2-phenylindole (Beyotime, Shanghai, China), and observed under the BX53 fluorescence microscope (×400) (Olympus, Japan).

### 2.7. Western Blotting

The radio-immunoprecipitation assay lysis buffer (Beyotime) containing protease inhibitors (Sigma-Aldrich) was mixed with cells or EVs, dissolved on ice for 30 minutes, and followed by centrifugation and supernatant collection. The protein concentration was determined by BCA kits (Pierce, IL, USA). Subsequently, the proteins were separated by 10% SDS-PAGE and electrically transferred onto polyvinylidene fluoride membranes. Then the membranes were placed in 5% skim milk prepared by Tris-buffered saline-tween (TBST), shaken and sealed for 1 hour to block the nonspecific binding. Afterwards, the membranes were incubated with primary antibodies anti-CD9 (ab236630, 1 : 1000, Abcam, Cambridge, UK), anti-CD81 (ab109201, 1 : 1000, Abcam), Anti-Calnexin (ab133615, 1 : 1000, Abcam), anti-*α*-SMA (ab124964, 1 : 1000, Abcam), anti-FAP-*α* (ab207178, 1 : 1000, Abcam), and anti-glyceraldehyde-3-phosphate dehydrogenase (GAPDH) (ab181602, 1 : 10000, Abcam) at 4°C overnight. The membranes were rinsed thrice with TBST for 5 minutes each and then probed with horseradish peroxidase-labeled secondary antibody (ab6721, 1 : 2000, Abcam) for 1 hour. Finally, the bands were developed using an enhanced chemiluminescence kit (Pierce). ImageJ software (Version 1.48, NIH, Bethesda, MD, USA) was utilized to quantify the gray values of each band, with GAPDH as an internal reference.

### 2.8. Enzyme-Linked Immunosorbent Assay (ELISA)

The levels of inflammatory cytokines IL-1*β* (ab214025, Abcam), IL-6 (ab178013, Abcam), and IL-8 (ab214030, Abcam) were measured using the corresponding kits.

### 2.9. 3-(4,5-Dimethylthiazol-2-yl)-2,5-Diphenyltetrazolium Bromide (MTT) Assay

The cell viability was measured using the MTT kits (M1020, Solarbio, Beijing, China), and the optical density value was measured at 490 nm on a microplate reader (Bio-Tek Instruments, VT, USA).

### 2.10. Cell Counting Kit-8 (CCK-8) Assay

Cells were seeded in 96-well plates at 2000/well, and cell proliferation was examined at 0, 6, 12, and 24 h using the CCK-8 kits. Experimental operations were carried out strictly under the kit instructions.

### 2.11. Transwell Assay

A 6.5 mm Transwell chamber (Costar, Jiangsu, China) with an aperture of 8 *μ*m was applied for the transwell invasion assay following the manufacturer's instructions. Briefly, Matrigel (YB356234, Yu Bo Biotech, Shanghai, China) stored at -80°C was melted at 4°C overnight. Next, Matrigel (200 *μ*L) was added to 200 *μ*L serum-free medium at 4°C for complete dilution. Then, 50 *μ*L of Matrigel was incubated in the apical chamber at 37°C for 2-3 hours. A549 cells (1 × 10^5^) were cultured in a serum-free medium to prepare cell suspension. Cell suspension (200 *μ*L) was paved on the apical chamber, and 800 *μ*L of cell suspension containing 10% FBS was added to the basolateral chamber for 24 hours. After that, the transwell plate was removed, washed twice with PBS, soaked in formaldehyde for 10 minutes, and rinsed with water 3 times. The cells stained with 0.5% crystal violet (Sigma-Aldrich) were left at room temperature for 30 minutes, and the cells in the upper surface were discarded with cotton balls. Later, the cells were observed and photographed with an inverted microscope (IX53, Olympus) and counted using the ImageJ software. Matrigel was not used in the transwell migration experiment, and cells were incubated for 24 hours. At least 4 areas were randomly selected for cell counting under the microscope.

### 2.12. Scratch Test

A549 cells were seeded into 6-well plates, and scratches were made in the center of the slide with a 200 *μ*L sterile pipette tip when the cells grew to about 2 × 10^6^/well. After 24 hours, the remaining cell-free area was measured and compared with the initial scratched area (in percentage). Images were acquired using a microscope (Zeiss, Germany), and the wound healing was analyzed using IncuCyte software (Essen BioScience, USA) to quantify cell migration.

### 2.13. Establishment of Nude Mouse Models

A total of 48 BALB/c nude mice (weighing 18 ± 2 g/mouse, aged 6-8 weeks) were purchased from Cavens Biogle Model Animal Research (Suzhou, China). To ensure that the experimental mice purchased were healthy, we followed the principles: (1) general conditions: good development, bright eyes, flexible response, free movement, good appetite, no congestion in the conjunctiva, no secretion in the pupil, no nasal agitation, sneezing, and scratching the cheek. (2) Fur color: clean, soft, glossy, no hair loss, fluffy, and fungal infection. (3) Abdominal respiration: the abdominal breathing of mice was even, without abdominal swelling. (4) External genitals: no damage, no purulent pain, and no odorous sticky secretions. (5) Characteristics of claw toe: no bite, no ulcer, and no scab.

All BALB/c mice were fed in a standard animal house with free drinking water and a diet at 24 ± 1°C with a humidity of 30%-40% for 1 week. They were kept under 12 hours of light/dark conditions with the light cycle from 8 : 00 to 20 : 00. A549 cells (2 × 10^6^) were injected into nude mice via the tail vein, with untreated A549 cells (2 × 10^6^) as the control group. Eight weeks later, mice were euthanized with pentobarbital sodium (100 mg/kg) followed by weighing lung tissue and counting metastatic nodules. Afterwards, lung tissues of 6 mice were embedded in paraffin, and lungs of 6 mice were homogenized into tissues and then stored at -80°C.

The mice were grouped as follows: the control group (injected with A549 cells), the NFs group (injected with A549 cells cultured in NFCM), the GW group (injected with A549 cells cultured in H358-GW-treated NFCM), and the EVs group (injected with A549 cells cultured in H358-EVs-treated NFCM).

### 2.14. Reverse Transcription Quantitative Polymerase Chain Reaction (RT-qPCR)

Total RNA was extracted from cells and tissues using the TRIzol reagent (Invitrogen) and reversely transcribed into cDNA using the PrimeScript RT reagent kits (Takara, Dalian, China). The TaqMan primers and probes used for detection were all from Takara. RT-qPCR was performed using ABI PRISM 7900 sequence detection system of SYBR Green II (Takara). PCR reaction conditions: predenaturation at 95°C for 5 minutes and 40 cycles of denaturation at 95°C for 15 seconds, annealing at 60°C for 20 seconds, and extension at 72°C for 35 seconds. With GAPDH as an internal reference, the data were analyzed with the 2^−ΔΔCt^ method. Primer sequences (synthesized by Sangon Biotech, Shanghai, China) are shown in Table 1 [46].

### 2.15. Hematoxylin-Eosin (HE) Staining

After routine dewaxing and hydration, paraffined sections were stained with hematoxylin, rinsed with running water, and differentiated with 0.7% ethanol hydrochloride. Next, the sections turned blue for about 15 minutes, immersed in 95% ethanol for 30 seconds, stained with eosin-containing ethanol for 30 seconds, soaked in gradient ethanol, cleared with xylene carbonate, sealed with neutral gum, and scanned with TissueFAXS (Tissuegnosti). The metastatic load was calculated as a percentage of tumor area to lung areas.

### 2.16. Immunohistochemistry

After dewaxing and hydration, the anti-Ki-67 antibody (Cat# M7240, Dako, Glostrup, Denmark) was used for immunohistochemical detection on the slides using the immunohistochemical kit (YDDEF001, Yuduo Biotech, Shanghai, China). Ki-67 was positive with brown-yellow granules in the nucleus. The number of Ki-67-positive tumor cells in 5 fields was calculated under a light microscope and averaged.

### 2.17. Statistical Analysis

GraphPad Prism 8.01 (GraphPad Software Inc., CA, USA) statistical software was used for statistical analysis and plotting of data. Graphics were typeset and drawn using Adobe Illustrator CC 2018 (Adobe Systems Incorporated, CA, USA). Data were expressed as mean ± standard deviation (SD). The *t*-test was used for data comparison between two groups, one-way analysis of variance (ANOVA) was used for data comparison among multiple groups, and Tukey's test was used for the post hoc test. *P* < 0.05 was considered statistically significant.

## 3. Results

### 3.1. T-EVs Promoted CAFs Activation

It has been reported that cancer cells stimulate mesenchymal fibroblasts through EVs in the TME and induce the activation of CAFs [47, 48]. We first cultured LC cells H358, normal lung epithelial cell line BEAS-2B, and lung NFs *in vitro,* and isolated EVs from H358 and BEAS-2B cell culture medium, respectively. EVs were “cup-shaped” under the TEM (Figure 1(a)). NTA showed that the particle size distribution of EVs ranged from 30 nm to 100 nm (Figure 1(b)). The protein levels of positive markers CD9 and CD81 and negative marker Calnexin on EV surface were examined by Western blotting, which manifested that compared to the GW (H358-GW/BeAS-2B-GW) group, CD9 and CD81 in EVs (H358-EVs/BeAS-2B-EVs) group were positive, while Calnexin was negative (Figure 1(c)). In addition, EVs labeled with red fluorescent dye Dil were cocultured with NFs. After 24 hours, immunofluorescence assay revealed that EVs (H358-EVs/BEAS-2B-EVs) were internalized by NFs (Figure 1(d)). EVs were successfully isolated and obtained, and NFs could internalize EVs (H358-EVs/BEAS-2B-EVs). Subsequently, the isolated EVs (H358-EVs/BEAS-2B-EVs) were cocultured with NFs. The protein levels of *α*-SMA and FAP-*α* on the surface of CAFs were measured by Western blotting, and levels of IL-1*β*, IL-6, and IL-8 were determined by ELISA. The results displayed that the protein levels of *α*-SMA and FAP-*α* as well as the levels of IL-1*β*, IL-6, and IL-8 in the EVs^H358^ group were significantly higher than those in the GW^H358^ group and theEVs^BEAS-2B^ group (*P* < 0.01), while there was no statistical difference among the NFs group, the GW^BEAS-2B^ group, the EVs^BEAS-2B^ group, and the GW^H358^ group (*P* > 0.05) (Figures 1(e) and 1(f)). Taken together, H358 cell-derived EVs accelerated the activation of CAFs.

### 3.2. T-EVs Promoted the Invasion and Migration of LC Cells through CAFs Activation

Studies have reported that CAFs regulate the TME by secreting a large number of proinflammatory factors (such as IL-6) and chemokines, thus enhancing the migration potential of LC cells [30, 48]. To further investigate whether H358-EVs can facilitate the invasion and migration of LC cells by inducing CAFs activation, the A549 cells were cultured in NFCM treated with EVs. MTT assay uncovered that relative to the GW^BEAS-2B^ group, the EVs^BEAS-2B^ group had high cell viability (*P* < 0.05), and the cell viability of the A549+EVs^H358^ group was visibly higher than that of the A549+GW^H358^ group and the EVs^BEAS-2B^ group (all *P* < 0.01) (Figure 2(a)). CCK-8 assay illustrated that the cell proliferation of the EVs^BEAS-2B^ group was greater than that of the GW^BEAS-2B^ group (*P* < 0.05), and the cell proliferation ability of the A549+EVs^H358^ group was stronger than that of the A549+GW^H358^ group or the EVs^BEAS-2B^ group (*P* < 0.01) (Figure 2(b)). Transwell assays and scratch tests illustrated that the EVs^BEAS-2B^ group had increased invasion and migration relative to the GW^BEAS-2B^ group (*P* < 0.05); compared to the A549+GW^H358^ group or the EVs^BEAS-2B^ group, the invasion and migration in the A549+GW^H358^ group were enhanced (all *P* < 0.01) (Figures 2(c)–2(e)). These results suggested that T-EVs can accelerate the invasion and migration of LC cells through CAFs activation.

### 3.3. H358-EVs Carried HOTAIR into NFs

LncRNA HOTAIR is highly expressed in LC [21, 40], and inhibition of HOTAIR can inhibit the growth of LC cells [43]. To elucidate whether H358-EVs carried HOTAIR into NFs, we first detected HOTAIR levels in H358 and BeAS-2B cells and the derived EVs by RT-qPCR. The results illustrated that HOTAIR levels in H358 cells and H358-EVs were significantly higher than those in BEAS-2B cells and BEAS-2B-EVs (all *P* < 0.01) (Figures 3(a) and 3(b)). H358-EVs were subsequently treated with Rnase and SDS, and no significant changes were discovered in HOTAIR levels after Rnase treatment (*P* > 0.05); however, HOTAIR level was lowered after treatment with Rnase and SDS simultaneously (*P* < 0.01) (Figure 3(b)). The above results suggest that HOTAIR was encapsulated in H358-EVs. Finally, after H358-EVs (50 *μ*g) were cocultured with NFs for 6 hours, HOTAIR level was visibly elevated (*P* < 0.01) (Figure 3(c)). In short, H358-EVs delivered HOTAIR into NFs.

### 3.4. H358-EVs Motivated the Activation of CAFs by Delivering HOTAIR

To further investigate whether H358-EVs promoted the activation of CAFs through HOTAIR transmission, EVs were isolated and extracted from H358 cells transfected with HOTAIR shRNA and cocultured with NFs for 6 hours. RT-qPCR showed that HOTAIR levels in H358 cells, and H358-EVs were reduced after treatment with HOTAIR shRNA (*P* < 0.01) (Figures 4(a) and 4(b)). Further detection showed lower HOTAIR levels in the EVs^H358-si-HOTAIR^ group than the EVs^H358-si-NC^ group (*P* < 0.01) (Figure 4(c)). Subsequently, Western blotting exhibited decreases in *α*-SMA and FAP-*α* protein levels in the EVs^H358-si-HOTAIR^ group relative to the EVs^H358-si-NC^ group (*P* < 0.01) (Figure 4(d)). ELISA showed that the levels of IL-1*β*, IL-6, and IL-8 in the EVs^H358-si-HOTAIR^ group were lower than those in the EVs^H358-si-NC^ group (*P* < 0.01) (Figure 4(e)). In summary, inhibition of HOTAIR expression in EVs partially averted the promotion effect of H358-EVs on CAFs activation, and H358-EVs expedited CAFs activation through HOTAIR transmission.

### 3.5. HOTAIR Downregulation Partially Annulled the Promotion Effects of H358-EVs-Mediated CAFs Activation on the Growth of LC Cells

The A549 cells were further cultured in NFCM treated with H358-EVs-si-HOTAIR followed by assessment of cell invasion and migration 24 hours later. After culture in H358-EVs-si-HOTAIR-treated NFCM, the cell viability was limited (*P* < 0.01) (Figure 5(a)), the cell proliferation was reduced (*P* < 0.05) (Figure 5(b)), and the invasion and migration were decreased (all *P* < 0.05) (Figures 5(c)–5(e)). To conclude, suppression of HOTAIR partially reversed the accelerating effect of H358-EVs-mediated CAFs activation on the invasion and migration of LC cells.

### 3.6. T-EVs Motivated Metastasis of LC *In Vivo* by Activating CAFs

To validate the effect of H358-EVs-mediated CAFs activation on LC metastasis *in vivo*, A549 cells (2 × 10^6^) were injected into nude mice. After 8 weeks, no prominent difference was observed in lung tissue weight and tumor nodules among the control group, NFs group, and GW group (*P* > 0.05), while these two indicators were higher in the EVs group than the GW group (*P* < 0.01) (Figures 6(a) and 6(b)). HE staining uncovered that a large number of tumor foci were formed in the lung of the EVs group, which was observably more than that of the GW group, accompanied by epithelial cell damage and disordered lamellar or fibrous arrangement of tumor cells. No statistical difference was found among the control group, NFs group, and GW group (Figure 6(c)). Immunohistochemistry exhibited more Ki-67-positive cells in lung tissues in the EVs group than that in the GW group (*P* < 0.01), whereas there was no prominent difference in Ki-67-positive cells in the control group, NFs group, and GW group (*P* > 0.05) (Figure 6(d)). Finally, RT-qPCR revealed a higher level of HOTAIR in lung tissues in the EVs group than that in the GW group (*P* < 0.01) and no evident difference in the control group, NFs group, and GW group (*P* > 0.05) (Figure 6(e)). Overall, T-EVs can promote LC metastasis *in vivo* by stimulating CAFs.

## 4. Discussion

LC is a common cancer with poor prognoses [49]. A recent study indicated that EVs can achieve molecular exchange between cancer cells and stromal cells, reshape local TME, and provoke tumorigenesis, development, and distant metastasis [49]. EVs contain abundant lncRNAs, and their interactions are essential in cell-to-cell information exchange [50]. CAFs, as activated fibroblasts in the tumor stroma, are known to promote cancer progression by altering the primary TME [51]. Our findings demonstrated that T-EVs carried HOTAIR into NFs and encouraged the activation of CAFs, thus promoting the invasion and metastasis of LC.

It has been acknowledged that communication networks mediated by EVs in the TME are critical in tumor development [52]. Specifically, T-EVs activate NFs to form a CAF-like phenotype and maintain a pro-TME [53]. Moreover, *α*-SMA and FAP are markedly expressed in CAFs and are regarded as surface markers of CAFs [54]. By expressing proinflammatory cytokines such as IL-1*β*, IL-6, and IL-8, CAFs regulate the inflammatory microenvironment [27, 29]. Firstly, LC cells (H358), normal lung epithelial cell line (BEAS-2B), and NFs were cultured *in vitro*, and EVs were extracted and identified. We found NFs could internalize EVs and the levels of CAFs surface markers (*α*-SMA/FAP-*α*) and cytokines (IL-1*β*/IL-6/IL-8) in T-EVs-treated NFs were elevated. These results strongly support the promoting effect of LC cell-derived EVs on CAFs activation. CAFs are actively recruited during cancer progression to support and promote tumor progression by secreting cytokines and growth factors [55]. Hence, LC cells A549 were cultured in H358-EVs-treated NFCM. Not surprisingly, A549 cells exhibited significant increases in cell viability, proliferation, invasion, and migration. In line with our findings, T-EVs motivate the activation of CAFs and accelerate the invasion of ovarian cancer [45]. Altogether, the aforementioned findings highlighted that T-EVs expedite the invasion and migration of LC cells by promoting CAFs activation.

EVs have been reported to deliver functional proteins, mRNAs, lncRNAs, and miRs to recipient cells [56, 57]. LncRNAs are critical players in the invasion and metastasis of LC [58]. In particular, lncRNAs carried by tumors participate in the activation of CAFs [21, 32]. Importantly, lncRNA HOTAIR level is upregulated in LC [21, 40]. Similarly, our findings revealed overexpressed HOTAIR levels in LC cells and their derived EVs, and HOTAIR was encapsulated in T-EVs. Moreover, the level of HOTAIR in T-EVs-treated NFs was substantially increased. Briefly, T-EVs transferred HOTAIR into NFs. Abnormal expression of lncRNAs in T-EVs induces NFs differentiation into CAFs, which plays a vital role in tumorigenesis [21, 32]. Given the abnormal expression of exosomal HOTAIR, we explored its role in the biological processes of LC cells. Subsequent experimentation in our study revealed that the knockdown of HOTAIR in EVs partially averted the promotive effects of T-EVs on CAFs stimulation and LC cell growth. Consistently, the knockout of HOTAIR inhibits CAF-induced tumor growth and lung metastasis *in vivo* [59]. In short, HOTAIR silencing partially reversed the promotion of T-EVs-mediated-CAFs activation on LC cell invasion and migration.

Finally, the metastasis of LC *in vivo* was analyzed by establishing nude mouse models. The high expression of Ki-67 is associated with the prognosis and clinicopathological features of LC patients [60]. We observed significant lung tissue damage in mice after injection of A549 cells cultured in H358-EVs-treated NFCM. Moreover, the number of Ki-67-positive cells in mouse lung tissue was markedly enhanced, suggesting that the tumor is prone to recurrence and metastasis. Besides, HOTAIR levels in mouse lung tissues were raised. Guo et al. demonstrated that CAFs-EVs promote the growth and metastasis of lung squamous cell carcinoma through *in vivo* tumor formation and metastasis experiments [61]. On the other hand, tumor-derived exosomal miR-1247-3p induces CAF activation to promote lung metastasis of hepatocellular carcinoma [48]. In light of the preceding literature, we concluded that T-EVs encouraged LC metastasis *in vivo* by activating CAFs.

In conclusion, we cultured A549 cells in NFCM treated with LC cell-derived EVs and verified that T-EVs induced the activation of CAFs by carrying HOTAIR, thus promoting the invasion and metastasis of LC. However, other molecular mechanisms of EVs promoting CAFs activation have not been described. Moreover, in addition to lncRNAs, T-EVs carry many other substances, such as proteins and miRNAs, which have very complex effects on the activation of CAFs, and these will be the direction of our further research in the future.

## Figures and Tables

**Figure 1:** T-EVs promoted CAFs activation. EVs were isolated from LC cell H358 and normal lung epithelial cell line BEAS-2B. (a) The morphology of EVs was observed by TEM; (b) NTA analysis of particle size distribution; (c) the expression of positive markers CD9 and CD81 and negative marker Calnexin on EV surface were detected by WB. EVs were labeled with red fluorescent dye Dil and cocultured with NFs; (d) the internalization of EVs by NFs was detected by immunofluorescence; (e) the protein levels of *α*-SMA and FAP-*α* on the surface of CAFs were detected by WB; and (f) the levels of cytokines IL-1*β*, IL-6, and IL-8 were detected by ELISA. Cell experiment was repeated three times. One-way ANOVA was used for data comparison among multiple groups in Figures (e) and (f), and Tukey's test was used for the post hoc test. ^∗∗^*P* < 0.01.

**Figure 2:** T-EVs promoted the invasion and migration of LC cells through CAFs activation. A549 cells were cultured in EVS-treated NFCM for 24 hours. (a) Cell viability was detected by MTT assay; (b) cell proliferation was detected by CCK-8 assay; (c, d) transwell assay was used to detect cell invasion and migration; (e) the scratch test was used to detect cell migration. Cell experiment was repeated three times. One-way ANOVA was used for data comparison among multiple groups, and Tukey's test was used for the post hoc test. ^∗^*P* < 0.05, ^∗∗^*P* < 0.01.

**Figure 3:** H358-EVs carried HOTAIR into NFs. RT-qPCR was adopted to detect the HOTAIR levels in H358 and BEAS-2B cells. (a) H358-EVs treated with Rnase and SDS. (b) H358-EVs (50 *μ*g) cocultured with NFs for 6 hours. (c) Cell experiment was repeated three times. The *t*-test was used for data comparison between groups in Figures (a)–(c), one-way ANOVA was used for data comparison among multiple groups in Figure (b), and Tukey's test was used for the post hoc test. ^∗∗^*P* < 0.01.

**Figure 4:** H358-EVs promoted the activation of CAFs by delivering HOTAIR. After transfection of H358 cells with HOTAIR inhibitor, EVs isolated and extracted were cocultured with NFs for 6 hours. (a–c) The levels of HOTAIR in H358 cells, EVs, and NFs were detected by RT-qPCR; (d) the protein levels of *α*-SMA and FAP-*α* on the surface of CAFs were detected by WB; (e) the levels of cytokines IL-1*β*, IL-6, and IL-8 were detected by ELISA. Cell experiment was repeated three times, and the *t*-test was used for data comparison between groups. ^∗∗^*P* < 0.01.

**Figure 5:** Inhibition of HOTAIR partially reversed the promotion of H358-EVs-mediated CAFs activation on invasion and migration of LC cells. A549 cells were cultured in NFCM treated with H358-EVs-si-HOTAIR for 24 hours. (a) Cell viability was detected by MTT; (b) cell proliferation was detected by CCK-8; (c, d) transwell assay was used to detect cell invasion and migration; (e) cell migration was detected by scratch test. Cell experiment was repeated three times. Repeated measures ANOVA was used for data comparison between groups in Figure (b), and *t*-test was used for data comparison between groups in Figures (a), (c), (d), and (e). ^∗∗^*P* < 0.01.

**Figure 6:** T-EVs promoted metastasis of LC *in vivo* by activating CAFs. A549 cells (2 × 10^6^) of each group were injected into nude mice via the tail vein. After 8 weeks, (a) The lung tissue was weighted, *N* = 12; (b) the number of tumor nodules was counted, *N* = 12; (c) HE staining was used to detect tumor foci in lung tissue, *N* = 6; (d) Ki-67-positive cells were detected by immunohistochemistry, *N* = 6; and (e) RT-qPCR was used to detect HOTAIR levels in lung tissues, *N* = 12. One-way ANOVA was used for data comparison among multiple groups, and Tukey's test was used for the post hoc test. ^∗∗^*P* < 0.01.

**Table 1:** Primer sequences.

Gene	Forward 5′-3′	Reverse 5′-3′
HOTAIR	GGCAAATGTCAGAGGGTT	GTGTAACAGGCAGGTGGA
GAPDH	CGCTGAGTACGTCGTGGAGT	CGTCAAAGGTGGAGGAGTGG

## Data Availability

The data in this study are available from the corresponding authors.
